The article "The Effect of Acute Kidney Injury on TGF-β1 and Smad3 in Patients with Coronary Heart Disease after Off-Pump Coronary Artery Bypass Grafting" was retracted in 2023. Reason: concerns about the peer review.

# The Effect of Acute Kidney Injury on TGF-*β*1 and Smad3 in Patients with Coronary Heart Disease after Off-Pump Coronary Artery Bypass Grafting

**DOI:** 10.1155/2021/1361242

**Published:** 2021-11-09

**Authors:** Shu Xu, Deng-shun Tao

**Affiliations:** Department of Cardiovascular Surgery, General Hospital of Northern Theater Command, Shenyang 110016, China

## Abstract

**Background:**

Acute kidney injury (AKI) is one of the most common and serious complications for coronary disease (CAD) patients, suffering from coronary artery bypass surgery (CABG). AKI occurs in nearly 30% of cardiac surgery patients, including CABG patients, affecting renal function, prolonging hospitalization time, and increasing all-cause mortality. TGF-*β*1 and Smad3 are sensitive biomarkers in evaluating kidney function. Therefore, comparing the TGF-*β*1 and Smad3 levels between the AKI patients and non-AKI patients after CABG surgery might have an important significance for identifying the risk degree of AKI and applying effective preventive measures after CABG surgery.

**Objective:**

This study aims at comparing the TGF-*β*1 and Smad3 levels between the AKI patients and non-AKI patients after CABG surgery to identify the risk degree of AKI and apply effective preventive measures after CABG surgery in clinics.

**Materials and Methods:**

A total of 25 proper patients, diagnosed as coronary disease (CAD) and undergoing AKI after CABG, were selected as the AKI group. The 25 participants, who did not suffer from AKI after CABG, were recruited using the case-control matching method in SPSS 25.0 software as the non-AKI group. Also, corresponding surgical specimens (tissues) and samples of blood were collected from them. Histopathological analysis and immunofluorescent microscopy of lesion artery and kidney of patients, who have been treated with kidney transplants, were performed on surgical specimens to find the pathological and histological change difference between the two groups. RT-PCR and Western blot were conducted to quantify the levels of TGF-*β*1 and Smad3 expression in serum for the patients of AKI and non-AKI groups, respectively.

**Results:**

Serious renal fibrosis was noted in patients of the AKI group. In addition, by H&E staining of the lesion artery, severe histopathological changes including smooth muscles proliferation with endothelial cell infiltration, focal degeneration and disruptions, and less collagen accumulation were found in the lesion artery of patients from the AKI group. Higher levels of TGF-*β*1 and Smad3 were observed in serum of patients of the AKI group.

**Conclusion:**

: The increased levels of TGF-*β*1 and Smad3 in serum might be risk factors for triggering AKI for CAD patients undergoing CABG.

## 1. Introduction

The acute kidney injury (AKI) caused postoperation is usually known as the acute renal failure and is one of the most severe complications caused postcoronary artery bypass grafting (CABG) [1–3]. It is a clinical disorder characterized by a rapid depreciation of the excretory kidney activity, by assembling urea and creatinine and reduced urinary output [4]. Approximately 30% of patients with diverse severity form AKI after their CABG surgery and around 2% need the short-term dialysis [5].

The postoperative AKI is correlated with surged cases of short and long-term morbidity and mortality [6]. There are multiple risk factors here, where the analysis and pathogenesis are difficult; thus, it is moderately comprehended [7]. Therefore, to boost the detection and outcomes, there is a necessity for an exclusive definition of AKI for implementation, research, and public health, for which Kidney Disease: Improving Global Outcomes (KDIGO) specifications have been advocated [8].

Recent studies indicate that even a small growth of serum creatinine followed by CABG are individually linked with increased mortality [9, 10]. The off-pump coronary artery bypass (OPCAB) grafting terminates the necessity of cardiopulmonary bypass (CPB) and thus, is communicated to be linked with little incidence of AKI [11–16]. Depending on the existence of cardiopulmonary bypass (CPB), CABG might be categorized into on-pump and off-pump CABG. Generally, CPB is considered to be the risk element for AKI after CABG because CPB is linked with inflammatory responses, renal hypoperfusion, free hemoglobin, nonpulsatile flow, and hemodilution [17]. Although, the possibility of the off-pump approach that might enhance the effects of CABG is still a disputed subject, as multiple studies have.

A corrective strategy to reducing the consequences of AKI would be significant. As a result, multiple factors may contribute to the pathogenesis of AKI following cardiac operations, including impaired autoregulation caused by comorbidities and medication, decreased renal perfusion due to altered hemodynamics during the procedure, and a systemic inflammatory response triggered by a major operation [18, 19]. As a result, there are many risk factors for CSA-AK1 injuries that cannot be changed. As a result, the time between coronary angiography (CAG) and coronary artery bypass graft surgery (CABG) has been presented as a risk factor that may be altered. According to the American Heart Association's (AHA) CABG recommendations, an interval of surgery after the CAG may be recommended for individuals with preexisting renal impairment until the effects of radiographic contrast material on renal function can be assessed [20].

## 2. Materials and Methods

### 2.1. Patient Sampling

Patients were selected for the study randomly from November 2019 to April 2021 who suffered from acute kidney injury after off-pump coronary artery bypass grafting for treatment of coronary heart disease. A total of 25 patients were selected randomly who reported acute kidney injury and who had surgical specimens (tissues) and samples of blood available. Patients who did not report acute kidney injury after off-pump coronary artery bypass grafting were excluded from the study.

Patients selected were compared in terms of gender, age, and alcohol/smoking parameters. Blood samples were collected (4 ml) from the true radial artery after bypass grafting, postsurgery, and postreporting of acute kidney injury. 25 samples were collected as controlled where the patients did not report any kidney injury. Samples of blood were first centrifuged at 3000 × *g* for five minutes; thus, plasma was collected at −80°C.

The surgical tissue specimens were collected postsurgeries, which went for histopathological and immunofluorescent analyses. The size of the tissues collected was around 0.2–0.4 cm, collected by picking holes in the anterior wall of the aorta (ascending) from patients who received off-pump coronary artery bypass grafting. Tissues collected were stored at −80°C. The RT-PCR (real-time reverse transcription polymerase chain reaction) process was performed to collect protein, RNA, and supernatant fluids for detection of TGF-*β*1 and Smad3 levels. The patient profile and demographics are given in Table 1. Surgically removed specimens were collected from patients who underwent off-pump coronary artery bypass grafting. The samples were stored and evaluated for estimating Smad3 and TGF-*β*1 levels.

### 2.2. Ethics

Current study was performed following the Declaration of Helsinki which was duly approved by the IREC (Institutional Research Ethics Committee). Thereby, admitted patients also signed a consent form to be a part of this study.

### 2.3. Quantitative RT-PCR

DNase I was used to remove DNA contamination from RNA samples which were collected for reverse transcription processing. 2–5 *μ*g RNA from each sample was collected and reverse transcribed into cDNA. The first strand synthesis system from Invitrogen, SuperScript III, was used to transcribe cDNA according to the standard protocols.

### 2.4. Reagents

Supplements and cell culture medias, FBS (fetal bovine serum), DMEM, SMEM, ITS (insulin/transferrin/selenium), and Penicillin, were obtained from Sigma-Aldrich, USA, and collagenase *α*2 type was purchased from Thermo Fisher Scientific Inc., Waltham, MA, USA.

PMSF (phenylmethanesulfonyl fluoride), simvastatin, *β*-glycerol 3-phosphate, and protease inhibitor cocktail were obtained from Beijing Biosynthesis Biotechnology Co., Ltd., Beijing, China, and ECL reagent– (enhanced chemiluminescence) was purchased from Bioworld Technology Inc., Louis Park, MN, USA. LysoTracker Red DND-99 was bought from Eugene, OR, USA, and Baf-A1 and 3-MA from Santa Cruz Biotechnology Inc., Santa Cruz, CA, USA. All the reagents purchased and obtained were of CSR grade or even better quality. Human scrambled shRN and human ATG7 shRNA were obtained from Bioworld Technology Inc., Louis Park, MN, USA.

### 2.5. Antibodies

Rabbit anti-human Smad2/3 and phospho-Smad3 antibodies were obtained from Sigma-Aldrich. Rabbit anti-human/mouse/rat LC3*β* II was obtained from Cell Signaling (Danvers, USA).

Collagen 1*α*2 (goat anti-human), GAPDH (glyceraldehyde-3-phosphate dehydrogenase) (mouse anti-human), and rabbit anti-human fibronectin were obtained from Sigma-Aldrich. Secondary antibodies, horseradish peroxidase and fluorochrome conjugated, were obtained from Bioworld Technology Inc., Louis Park, MN, USA.

### 2.6. Immunohistochemistry

Tissues obtained were fixated in 95% ethanol solution. Isolated tissues kept at −80°C were used for sectioning. 7 *μ*M thick sections were cut from frozen tissue blocks along the scarred region by help of Microm HM 550 cryotome. The sections were placed on slides, fixed for 15 minutes in a solution of 4% paraformaldehyde, followed by 3 items of washing in 1% PBS buffer solution, and finally fixed with 0.1% triton for 15 minutes duration.

The tissue slices were washed 3 times for 15 minutes in a PBS solution (1%). Tissues were then incubated at 4°C by using antibodies (primary) in a bovine serum albumin solution 1%. Slices of tissues were thoroughly washed at 3 × 15 min next day with PBS (1%) solution. Tissues were again incubated at room temperature for 90 minutes with secondary antibodies fluorescently conjugated. Washing of slides was repeated with 1% PBS for 3x for 15 min and then dried. Prolong Gold antifade reagent from Thermo Fisher Scientific Inc. was used to mount the slides' coverslips with DAPI. The fluorescence microscope was used to capture Invitrogen EVOS M7000 (Thermo Fischer EVOS Imaging) images with ×40 magnification.

### 2.7. Statistical Analysis

The results expressed are mean ± SEM, where the statistical differences were also determined using two-way ANOVA and Tukey's post hoc test. *P* value of 0.05 is considered significant. Three times collection of data was done for cell cultures separately.

## 3. Results

Symptoms including oliguria and backache and abnormal serum nitrogen and creatinine levels were found for all patients in the AKI group. The renal function stage distributions represented as the glomerular filtration rate (GFR) for patients in the AKI group are given in Table 1.

Serious renal fibrosis was noted in patients of the AKI group who have been treated with kidney transplants. It is presented in the renal specimens of sample subjects A and B, as shown in Figure 1.

TGF-*β*1 and Smad2 were expressed heavily in the kidney essence and proved in the renal specimens of sample subjects A and B by immunohistochemical staining, as shown in Figure 2.

H&E staining of the lesion artery showed severe histopathological changes including smooth muscles proliferation with endothelial cell infiltration (Figure 3(a)), focal degeneration and disruptions (Figure 3(b)), and less collagen accumulation (Figure 3(c)) in patients from the AKI group. Also, the result has been confirmed in lesion artery specimens of patients from AKI and non-AKI groups with obviously higher expressions of TGF-*β*1 and Smad3 by Western blot detection, as shown in Figure 4.

Compared with the patients in the non-AKI group by ELISA detection, the levels of TGF-*β*1 and Smad3 in serum of patients in the AKI group were significantly higher (non-AKI vs. AKI group: TGF-*β*1: 154.7 ± 33.6 vs 412.6 ± 62.8 ng/L, *t* = 18.10, *P* < 0.001; Smad3: 9.1 ± 3.8 vs 27.1 ± 5.2 ng/L, *t* = 13.97, *P* < 0.001), as shown in Figure 5.

## 4. Discussion and Conclusion

The levels of TGF-*β*1 and Smad3 were significantly increased in CAD patients with acute kidney injury. The serum levels of TGF-*β*1 and Smad3 were lower in control groups. Fibrosis was also noted in renal tissues collected from the patients suffering from renal injury. The immunofluorescent images also showed high levels of TGF-*β*1 and Smad3 in the injury group when compared against no renal injury control groups. Histopathological examination of radial artery tissues stained with eosin and hematoxylin revealed minor abnormalities in cell infiltration and localized degeneration. Following off-pump grafting, collagen accumulation was also observed in the vascular regions. Deep fibrosis in the renal tissues was notably documented as a cause of kidney injury, thus supporting the kidney damage after grafting. TGF-*β*1 and Smad3 have a prominent role to play in intensifying the damage postgrafting in CAD patients. Hence, it is concluded that TGF-*β*1 and Smad3 are strongly correlated to CAD and their further increase leads to acute kidney injuries, thus increasing the chances of renal problems postgrafting in patients.

## Figures and Tables

**Figure 1:** Serious renal fibrosis in patients of the AKI group. H&E staining of kidney specimens from sample subjects A and B who have been treated with kidney transplants.

**Figure 2:** TGF-*β*1 and Smad2 expressed heavily in the kidney essence in patients of the AKI group. Immunohistochemical staining of kidney specimens from sample subjects A and B, who have been treated with kidney transplants.

**Figure 3:** H&E staining of the lesion artery showing histopathological changes including smooth muscles proliferation with endothelial cell infiltration (a), lesion artery focal degeneration and disruptions (b), and less collagen accumulation (c) in patients from the AKI group.

**Figure 4:** Expressions of TGF-*β*1 and Smad3 in lesion artery specimens of patients from non-AKI and AKI groups.

**Figure 5:** The levels of TGF-*β*1 and Smad3 in serum of the patients in the non-AKI group and AKI group.

**Table 1:** Renal function distributions for patients in the AKI group.

Stages	Renal functioning	Patients (proportion, %) in the AKI group
I	GFR >89 mL/min	3 (12)
II	GFR 60–89 mL/min	12 (48)
III	GFR 30–59 mL/min	9 (36%)
IV	GFR 15–29 mL/min	1 (4)

## Data Availability

The data used to support the results of the study are available from the first author or corresponding author upon request.

## Abbreviations

RA: Radial artery
TGF-*β*1: Transforming growth factor-*β*1
AKI: Acute kidney injury
CABG: Coronary artery bypass grafting
GAPDH: Glyceraldehyde-3-phosphate dehydrogenase
GFR: Glomerular filtration rate
PBS: Phosphate buffered saline.

## References

[1] Loef B. G., Epema A. H., Smilde T. D. (2004). Immediate postoperative renal function deterioration in cardiac surgical patients predicts in-hospital mortality and long-term survival. *Journal of the American Society of Nephrology*.

[2] Rosner M. H., Okusa M. D. (2005). Acute kidney injury associated with cardiac surgery. *Clinical Journal of the American Society of Nephrology*.

[3] Ryckwaert F., Boccara G., Frappier J.-M., Colson P. H. (2002). Incidence, risk factors, and prognosis of a moderate increase in plasma creatinine early after cardiac surgery. *Critical Care Medicine*.

[4] Reents W., Hilker M., Börgermann J. (2014). Acute kidney injury after on-pump or off-pump coronary artery bypass grafting in elderly patients. *The Annals of Thoracic Surgery*.

[5] Ronco C., Bellomo R., Kellum J. A. (2019). Acute kidney injury. *The Lancet*.

[6] Coca S. G., Bushra Y., Shlipak M. G., Garg A. X., Parikh C. R. (2009). Long-term risk of mortality and other adverse outcomes after acute kidney injury: a systematic review and meta-analysis. *American Journal of Kidney Diseases*.

[7] Birch M., Lupei M., Weinkauf J. (2018). Long-term complications and management. *Kaplan’s Essentials of Cardiac Anesthesia*.

[8] Zhang Y., Nan Y., Chen Y.-P., Cheng H. (2013). Relation between the interval from coronary angiography to selective off-pump coronary artery bypass grafting and postoperative acute kidney injury. *The American Journal of Cardiology*.

[9] Brown J. R. (2006). Perioperative increases in serum creatinine are predictive of increased 90-day mortality after coronary artery bypass graft surgery. *Circulation*.

[10] Lassnigg A. (2004). Minimal changes of serum creatinine predict prognosis in patients after cardiothoracic surgery: a prospective cohort study. *Journal of the American Society of Nephrology*.

[11] Hix J. K., Thakar C. V., Katz E. M., Yared J.-P., Sabik J., Paganini E. P. (2006). Effect of off-pump coronary artery bypass graft surgery on postoperative acute kidney injury and mortality. *Critical Care Medicine*.

[12] Sajja L. R., Mannam G., Chakravarthi R. M. (2007). Coronary artery bypass grafting with or without cardiopulmonary bypass in patients with preoperative non-dialysis dependent renal insufficiency: a randomized study. *The Journal of Thoracic and Cardiovascular Surgery*.

[13] Srinivasan A. K., Grayson A. D., Fabri B. M. (2004). On-pump versus off-pump coronary artery bypass grafting in diabetic patients: a propensity score analysis. *The Annals of Thoracic Surgery*.

[14] Stallwood M. I., Grayson A. D., Mills K., Scawn N. D. (2004). Acute renal failure in coronary artery bypass surgery: independent effect of cardiopulmonary bypass. *The Annals of Thoracic Surgery*.

[15] Weerasinghe A., Thanos A., Sharif Al-R. (2005). Functional renal outcome in on-pump and off-pump coronary revascularization: a propensity-based analysis. *The Annals of Thoracic Surgery*.

[16] Wijeysundera D. N., Beattie W. S., Djaiani G. (2005). Off-pump coronary artery surgery for reducing mortality and morbidity. *Journal of the American College of Cardiology*.

[17] Pickering J. W., James M. T., Palmer S. C. (2015). Acute kidney injury and prognosis after cardiopulmonary bypass: a meta-analysis of cohort studies. *American Journal of Kidney Diseases*.

[18] Abuelo J. G. (2007). Normotensive ischemic acute renal failure. *New England Journal of Medicine*.

[19] Schrier R. W., Wei W., Brian P., Amit M. (2004). Acute renal failure: definitions, diagnosis, pathogenesis, and therapy. *Journal of Clinical Investigation*.

[20] Hillis L. D., Smith P. K., Anderson J. L. (2011). 2011 ACCF/AHA guideline for coronary artery bypass graft surgery. *Journal of the American College of Cardiology*.

